RETRACTED

# Brain injury following cardiac arrest: pathophysiology for neurocritical care

**DOI:** 10.1186/s40560-016-0140-9

**Published:** 2016-04-27

**Authors:** Hiroyuki Uchino, Yukihiko Ogihara, Hidekimi Fukui, Miyuki Chijiiwa, Shusuke Sekine, Naomi Hara, Eskil Elmér

**Affiliations:** Department of Anesthesiology, Tokyo Medical University, 6-7-1 Nishishinjuku, Shinjuku-ku, Tokyo, 160-0023 Japan; Mitochondrial Pathophysiology Unit, Department of Clinical Sciences, Lund University, Box 117, 221 00 Lund, Sweden

**Keywords:** Pathophysiology of ischemic brain damage, Cardiac arrest, Post-cardiac arrest syndrome (PCAS), Mitochondrial dysfunction, Reperfusion injury, Excitotoxicity, Mitochondrial permeability transition (MPT), Calcineurin/immunophilin

## Abstract

Cardiac arrest induces the cessation of cerebral blood flow, which can result in brain damage. The primary intervention to salvage the brain under such a pathological condition is to restore the cerebral blood flow to the ischemic region. Ischemia is defined as a reduction in blood flow to a level that is sufficient to alter normal cellular function. Brain tissue is highly sensitive to ischemia, such that even brief ischemic periods in neurons can initiate a complex sequence of events that may ultimately culminate in cell death. However, paradoxically, restoration of blood flow can cause additional damage and exacerbate the neurocognitive deficits in patients who suffered a brain ischemic event, which is a phenomenon referred to as “reperfusion injury.” Transient brain ischemia following cardiac arrest results from the complex interplay of multiple pathways including excitotoxicity, acidotoxicity, ionic imbalance, peri-infarct depolarization, oxidative and nitrative stress, inflammation, and apoptosis. The pathophysiology of post-cardiac arrest brain injury involves a complex cascade of molecular events, most of which remain unknown. Many lines of evidence have shown that mitochondria suffer severe damage in response to ischemic injury. Mitochondrial dysfunction based on the mitochondrial permeability transition after reperfusion, particularly involving the calcineurin/immunophilin signal transduction pathway, appears to play a pivotal role in the induction of neuronal cell death. The aim of this article is to discuss the underlying pathophysiology of brain damage, which is a devastating pathological condition, and highlight the central signal transduction pathway involved in brain damage, which reveals potential targets for therapeutic intervention.

## Introduction

Out-of-hospital cardiac arrest (OHCA) is a common initial disease in developed countries. According to the latest report, of the 123,987 patients with OHCA in Japan brought to the hospital, 75,397 patients were suffering from a cardiogenic cause. The survival rate of the patients with bystander at 1 month was 11.9 % and the survival rate to hospital discharge was only 7.9 % (http://www.fdma.go.jp/neuter/topics/kyukyukyujo_genkyo/h26/01_kyukyu.pdf).

RETRACTED

Patients who achieve return of spontaneous circulation (ROSC) after OHCA show significant morbidity and mortality due to the cerebral and cardiac dysfunction that leads to prolonged whole-body ischemia. This syndrome, called the post-cardiac arrest syndrome (PCAS), comprises anoxic brain injury, post-cardiac arrest myocardial dysfunction, systemic ischemia/reperfusion response, and persistent precipitating pathology. Cardiac arrest is often associated with neurological deterioration. Although many years of laboratory and clinical research have been spent, post-cardiac arrest brain injury (PBI), a key factor of PCAS that involves complex molecular mechanisms, remains a common cause of morbidity and mortality. The four key components of PCAS were identified as (1) PBI, (2) post-cardiac arrest myocardial dysfunction, (3) systemic ischemia/reperfusion response, and (4) persistent precipitating pathology [1]. Many studies have examined the mechanisms involved in ischemic brain injury. However, no effective pharmacological treatment directed at tissues of the central nervous system (CNS) has been established to prevent the pathological conditions that occur as a consequence. Therefore, all aspects of the basic mechanisms responsible for brain damage require urgent elucidation. Recently, our research has aimed towards understanding the involvement and importance of calcium and the calcineurin/immunophilin signal transduction pathway in brain damage. We previously demonstrated that immunosuppressants interacting with the calcineurin/immunophilin signal transduction pathway show potent neuroprotective effects in several animal models of ischemic brain damage, and these effects are considered to be separate from their action on immunocompetent cells [2–6].

In clinical anesthesiology, the pathological conditions that involve neuronal degeneration can be broadly divided into several categories as follows: (i) global ischemia due to an extended period of cardiac arrest [7, 8]; (ii) cerebral infarction (focal ischemia) that occurs after the occlusion of cerebral arteries; (iii) direct injuries due to head trauma and cerebral compression associated with hematoma or cerebral edema; (iv) increased intracranial pressure and secondary hypoxic brain damage due to cerebrovascular spasm; (v) encephalitis or meningitis caused by viruses, bacteria, parasites, fungi, and spirochetes; and (vi) seizures caused by head trauma, cerebral tumors, cerebrovascular disorders, intracranial infections, and abnormal metabolism. This condition is likely to share many aspects of the pathological mechanisms resulting in brain damage and neurological impairment. Although the most crucial mechanisms responsible for the induction of brain damage remain unclear, it has been suggested that mitochondrial dysfunction is significantly involved. The elucidation of the basic pathophysiology for each of these pathological conditions that involve neuronal degeneration is of great importance for the development of effective neuroprotective pharmaceutical agents.

RETRACTED

In this review, we outline the role of major pathophysiological disturbances leading to PBI and PCAS due to cardiac arrest that involve increased intracellular calcium, reactive oxygen species (ROS), and inflammation in ischemic neuronal cell death, with special emphasis on the mitochondrial permeability transition (MPT), which is a pathological state of the inner mitochondrial membrane leading to bioenergetic failure [9–12].

## Review

### Pathophysiology of post-cardiac arrest brain injury and delayed neurodegeneration

At the onset of cardiac arrest, cerebral blood flow tends to approach zero. In response to the stress of global ischemia, various cytokines and complement anaphylatoxins are synthesized and released. During cardiopulmonary resuscitation (CPR), blood flow is partially restored. Optimal CPR can restore the cardiac output to between 25 and 40 % of pre-arrest values, while the brain receives 30 % of this amount [13]. After onset of reperfusion, the activation of blood coagulation leads to the formation of microemboli, while the activated neutrophils and platelets accumulate in microvessels [14]. Cerebral microvascular blood flow may further be compromised by the α1-adrenergic agonist action of endogenous or exogenous adrenaline which reduces capillary blood flow and increases arterial lactate levels [15]. During reperfusion, the generated ROS intensify endothelial injury, increasing the exchange vessel’s permeability and microvascular filtration [14].

After ROSC, a transient increase in circulating catecholamine concentrations results in a normal or elevated blood pressure immediately, and high pressure periods are needed to overcome the potential no-reflow phenomenon. Several cytokines, which directly inhibit adrenal cortisol synthesis and increase the risk of early refractory shock, are upregulated which promote tissue damage due to neutrophil infiltration [16]. The ATP-generating capacity of the mitochondria and energy charge of the tissue increase and are normalized after 1 h of reperfusion [17]. Lactate accumulation occurs during cardiac arrest and CPR; it is an essential aerobic energy substrate and contributes to neuronal integrity post-ischemia. Lactate is the main oxidizable energy substrate utilized by the brain, at least during the initial moments after ROSC.

RETRACTED

The conditions after ROSC favor the opening of the mitochondrial permeability transition pore (mtPTP) which is now characterized by non-specific permeabilization of the inner mitochondrial membrane, resulting in a dramatic swelling of the mitochondria, followed by disruption of the outer membrane, particularly in the reperfused tissues [10]. The opening of mtPTP activates processes that lead to a delayed neuronal death after 24–48 h of recovery.

The levels of various interleukins are intensely increased and reach their peak concentration in the blood approximately 3 h after ROSC, indicating a “systemic inflammatory response syndrome” [18] during the early post-arrest phase. The impact of ischemia/reperfusion injury on brain injury increases with aging [19]. The impairment of brainstem function in aged patients may further deteriorate, resulting in increased mortality and morbidity following cardiac arrest and resuscitation.

Pathophysiological disorders occur from the onset of cardiac arrest; however, the clinical manifestations of neuronal degeneration are delayed. Massive functional neurological impairment may occur after ROSC, and morphological changes in the brain reach maximum levels after 3 weeks. The pathogenesis of delayed neuronal injury is further complicated by the fact that it occurs even in successfully recirculated brains. The post-ischemic hypoperfusion syndrome may evolve due to the mismatch between blood flow and oxygen requirements of the tissue.

### Induction of ischemic neuronal cell death—the glutamate-Ca^2+^ theory

Ischemia is defined as a reduction in blood flow to a level that is sufficient to alter normal cellular function. Brain tissue is highly sensitive to ischemia, such that even brief ischemic periods in neurons can initiate a complex sequence of events that may ultimately culminate in cell death. Different brain regions have varying thresholds for ischemic cell damage, with the white matter being more resilient than the gray matter [1]. Discontinuation of aerobic metabolism due to cerebral ischemia provokes the immediate loss of energy substrates, promotes anaerobic glycolysis with the accumulation of intracellular lactic acid and H^+^, leading to intracerebral acidosis. Under conditions of hyperglycemia, intracerebral acidosis is exaggerated. Furthermore, there is a loss of energy-dependent ion homeostasis primarily caused by the inhibition of the plasma membrane ATP-dependent Na^+^/K^+^ exchanger, resulting in an increase in extracellular K^+^ as well as intracellular Na^+^, leading to cellular depolarization. The ion gradients that are normally established across the plasma membrane have many functions, for example, they are used for the removal of excess intracellular Ca^2+^ as well as for the re-uptake of extracellular glutamate. These functions are abolished during ischemia. Moreover, Ca^2+^ influx via voltage-dependent Ca^2+^ channels can contribute to the release of glutamate from presynaptic terminals to the extracellular space [20]. The excessive release of glutamate further provokes an increase in intracellular Ca^2+^ and Na^+^ levels by the binding of glutamate to its postsynaptic receptors (i.e., *N*-methyl-*D*-aspartate [NMDA] receptors and α-amino-3-hydroxy-5-methylisoxazole-4-propionic acid [AMPA] receptors). During ischemia, extracellular calcium concentration (Ca)e decreases abruptly from about 1.2 mM to about 0.2 mM, demonstrating that virtually all extracellular Ca^2+^ is taken up by cells [21–23]. This increase in intracellular Ca^2+^ and Na^+^ levels activates the signal transduction pathways mediated by the activation of Ca^2+^-dependent enzymes including nitric oxide synthase, phospholipase A2, and calmodulin kinase, which then trigger the following intracellular events: degradation of lipid membrane components, an increase in the levels of free fatty acids, alteration of gene expression, alteration of the phosphorylation and de-phosphorylation state of proteins, degradation of proteins of the cytoskeleton, enzymatic and mitochondrial production of free radicals such as ROS (e.g., superoxide, hydroxyl radicals, and hydrogen peroxide (H_2_O_2_)) or reactive nitrogen species (Fig. 1). In addition, the increased intracellular Ca^2+^ levels will trigger mitochondrial dysfunction (described separately below and in Fig. 2). This results in the deterioration of neuronal cell membranes and organelles, induction of downstream cascades involving increased Ca^2+^ cycling and Ca^2+^ overload (calcium dysregulation), activation of suicide programs, disturbance of axonal transport, activation of macrophages by the expression of adhesion factors, and platelet aggregation associated with microvascular dysfunction, which will eventually lead to unavoidable cell death (Fig. 3). Clinical manifestations of rapid or delayed neuronal degeneration may occur.

RETRACTED

**Fig. 1:** Pathophysiology of post-cardiac arrest syndrome. The four key components of PCAS were identified as (1) post-cardiac arrest brain injury, (2) post-cardiac arrest myocardial dysfunction, (3) systemic ischemia/reperfusion response, and (4) persistent precipitating pathology

**Fig. 2:** Relationship to the site of post-cardiac arrest care. Patients with ROSC receive >20-min care during transport or in the ED before hospital admission. The first 20 min after ROSC is defined as the immediate post-arrest phase. Between 20 min and 6–12 h after ROSC is defined as the early post-arrest phase. Between 6 and 12 and 72 h is defined as the intermediate phase. A period beyond 3 days is defined as the recovery phase when prognostification becomes more reliable (cited and modified from Noran 2009)

**Fig. 3:** Calcium overload and the calcineurin/cyclophilin D signal transduction pathway for the cell death induced after cerebral ischemia. Ischemia induces the loss of ATP-dependent ion homeostasis and leads to an increase in intracellular Na^+^ and extracellular K^+^. Eventually, the cells undergo depolarization. As a result, excessive Ca^2+^ influx due to the activation of voltage-sensitive calcium channels, NMDA, and AMPA receptors activates numerous signal transduction cascades, particularly the calcineurin/cyclophilin D signal transduction pathway. This eventually induces the MPT, leading to mitochondrial dysfunction

This glutamate-Ca^2+^ theory of excitotoxic neuronal cell death is widely accepted [24–26]. According to this theory, the most important aspect of the pathogenesis of cerebral ischemia is the restriction of substrates and oxygen to the mitochondrial respiratory system and the induction of cellular ATP crisis. It is the loss of cellular energy and its repercussions that trigger acute or delayed neuronal cell death. However, recent analyses of the role played by heart and liver mitochondria in reperfusion injury [27, 28] strongly indicate that direct calcium-triggered mitochondrial dysfunction and neuronal cell death associated with the induction of the MPT may be involved in reperfusion injury under situations of decreased cellular energy levels (lowered levels of ATP) and increased oxidative stress (Fig. 4). During the last 10 years, we have investigated and characterized the MPT in isolated mitochondria from the CNS as well as examined the role of inhibitors of the MPT in in vivo models of brain disease. The MPT is an exciting new putative therapeutic target for intervention in ischemia reperfusion injury [3, 8, 21, 29–36].

**Fig. 4:** Mitochondrial permeability transition and ischemic brain damage. Various forms of stress, such as brain ischemia, hypoxia, traumatic brain injury, status epilepticus, and encephalitis, induce mitochondrial dysfunction and the MPT that lead to apoptosis or necrosis. Calcineurin and immunophilin (CypD) are the key factors that induce the apoptotic pathway, and the immunosuppressants CsA and FK506 exert their neuroprotection by the inhibition of calcineurin and CypD activity

RETRACTED

### Post-cardiac arrest myocardial dysfunction

Post-cardiac arrest myocardial dysfunction also contributes to the low survival rate [37]; however, this phenomenon is both responsive to therapy and reversible [13, 38]. Heart rate and blood pressure are extremely variable due to the transient increase in local and circulating catecholamine concentrations after ROSC [39]. In one series of 148 patients who underwent coronary angiography after cardiac arrest, 49 % of the subjects had myocardial dysfunction manifested by tachycardia and elevated left ventricular end-diastolic pressure, followed approximately 6 h later by hypotension (MAP < 75 mmHg) and low cardiac output (cardiac index <2.2 L min^−1^ m^−2^) [13]. Several case series have described transient myocardial dysfunction after human cardiac arrest. Cardiac index values reached their nadir at 8 h after resuscitation, improved substantially by 24 h, and almost uniformly returned to normal by 72 h in patients who survived OHCA [13]. The responsiveness of post-cardiac arrest global myocardial dysfunction to inotropic drugs is well documented in animal studies [38, 40].

### Reperfusion injury and reactive oxygen species (ROS)

It is well known that reperfusion following brain ischemia induces the production of a large amount of ROS ubiquitously throughout a cell. Cardiac arrest represents the most severe shock state, during which delivery of oxygen and metabolic substrates is abruptly halted and metabolites are no longer removed. CPR only partially reverses this process, achieving cardiac output and systemic oxygen delivery (DO_2_) that is much less than normal. During CPR, a compensatory increase in systemic oxygen extraction occurs, leading to significantly decreased central (ScvO_2_) or mixed venous oxygen saturation [22]. The whole-body ischemia/reperfusion of cardiac arrest with associated oxygen debt causes generalized activation of immunological and coagulation pathways, increasing the risk of multiple organ failure and infection [23, 41, 42]. Activation of blood coagulation without adequate activation of endogenous fibrinolysis is an important pathophysiological mechanism that may contribute to microcirculatory reperfusion disorders [43, 44]. The stress of total body ischemia/reperfusion affects adrenal function. Although an increased plasma cortisol level occurs in many patients after OHCA, relative adrenal insufficiency, defined as failure to respond to corticotrophin (i.e., <9 μg mL^−1^ increase in cortisol), is common [45, 46]. Clinical manifestations of a systemic ischemic-reperfusion response include intravascular volume depletion, impaired vasoregulation, impaired oxygen delivery and utilization, and increased susceptibility to infection.

RETRACTED

A potentially devastating sequence of reperfusion events is one in which resumption of oxygen supply leads to grossly enhanced production of ROS and, thereby, leads to free radical-mediated damage. The restoration of cerebral blood flow, which is known as “reperfusion,” elicits multiple cellular and physiologic events. Reperfusion reverses the disruption of cellular functions that was induced by ischemia. In adults, ischemic insults to the brain typically result from stroke (caused by either thrombotic occlusion or rupture of a blood vessel) [47] or cardiac arrest [48], whereas in infants, cerebral ischemia can be initiated by complications during delivery, resulting in neonatal hypoxic-ischemic encephalopathy [49]. Spontaneous reperfusion or reperfusion created by an intervention can cause additional and substantial brain damage, which is referred to as “reperfusion injury.” Reperfusion induces pathological events such as lipid peroxidation due to the elevation of ROS, inflammation, and calcium overload (calcium dysregulation) that leads to MPT associated with mitochondrial dysfunction [27, 28, 50, 51] (further discussed below).

There are a number of possible cellular sources of these free radicals, including xanthine oxidase, cyclooxygenase, lipoxygenase, cytochrome p450, endothelial nitric oxide synthase, and NADPH oxidase. Mitochondria also produce ROS in the form of a superoxide anion (O^2−^), H_2_O_2_, and hydroxyl radical (OH^−^) which have been suggested to play important roles in the regulation of signal transduction and cellular metabolism [52]. Alterations of phosphorylating (state 3) and basal (state 4) respiration and respiratory control indicate a normalization of the electron transport system after reperfusion. However, secondary mitochondrial dysfunction is a prominent consequence of transient cerebral ischemia [53] resulting in a reduction of mitochondrial ATP synthesis. The other major target of ROS is lipids, and the peroxidative action of ROS promotes the inactivation of key metabolic enzymes that regulate glucose metabolism. ROS are inactivated by endogenous mitochondrial and cytoplasmic scavenging systems. However, ischemic reperfusion can sometimes overwhelm these scavenging systems, resulting in the production of ROS originating primarily from mitochondrial complexes I and III of the electron transport chain, causing oxidative damage to the mitochondria and consequently the cell [54]. Other highly reactive free radicals are produced by protein nitrosylation due to the reaction of NO and superoxide anions, which can also lead to the dysregulation of cellular homeostasis.

RETRACTED

### Persistent precipitating pathology

Diagnosis and management of persistent precipitating pathologies such as acute coronary syndrome (ACS), pulmonary diseases, hemorrhage, sepsis, and various toxic syndromes can complicate and be complicated by the simultaneous pathophysiology of PCAS. Consecutive patients had no obvious non-cardiac etiology but had undergone coronary angiography after resuscitation from OHCA [55]. Nine of the patients with acute coronary occlusion did not have chest pain or ST segment elevation. Elevations in troponin T measured during treatment of cardiac arrest suggest that ACS precedes OHCA in 40 % of the patients [56]. Another thromboembolic disease to consider after cardiac arrest is pulmonary embolism. Pulmonary emboli have been reported in 2–10 % of sudden deaths [57, 58].

Primary pulmonary diseases such as chronic obstructive pulmonary disease, asthma, or pneumonia can lead to respiratory failure and cardiac arrest. When cardiac arrest is caused by respiratory failure, pulmonary physiology may be worse after restoration of circulation. Redistribution of blood into pulmonary vasculature can lead to frank pulmonary edema or at least increased alveolar-arterial oxygen gradients after cardiac arrest [59]. Acute brain edema is more common after cardiac arrest caused by asphyxia [60]. It is possible that perfusion with hypoxemic blood during asphyxia preceding complete circulatory collapse is harmful.

Sepsis is a cause of cardiac arrest, acute respiratory distress syndrome, and multiple organ failure. Thus, there is a predisposition for exacerbation of PCAS when cardiac arrest occurs in the setting of sepsis. Other precipitating causes of cardiac arrest may require specific treatment during the post-cardiac arrest period. For example, drug overdose and intoxication may be treated with specific antidotes, and environmental causes such as hypothermia may require active temperature control.

### Disturbance of mitochondrial Ca^2+^ homeostasis in neurons

During ischemia, neuronal Ca^2+^ channels and transporters as well as glutamate receptors are overactivated, and the increased activity of plasma membrane Ca^2+^ channels can then trigger the entry of Ca^2+^ into the cytosol, leading to Ca^2+^ overload. Mitochondria contain two membranes, an outer membrane permeable to solutes and an inner membrane impermeable to solutes that harbors the respiratory chain complexes. Mitochondria powerfully sequester Ca^2+^ to prevent the elevation of cytosolic Ca^2+^, but prolonged depolarization and Ca^2+^ influx lead to mitochondrial Ca^2+^ overload. Mitochondrial Ca^2+^ overload is induced by three mechanisms: (i) increased mitochondrial Ca^2+^ uptake following the release of Ca^2+^ from the endoplasmic reticulum and Ca^2+^ influx from the extracellular space, (ii) reduced Ca^2+^ extrusion through the mitochondrial Na^+^/Ca^2+^ exchanger, and (iii) changes in the capacity of mitochondrial Ca^2+^ buffering [61]. Moderate increases in mitochondrial Ca^2+^ concentration are necessary and sufficient to adjust ATP production to cell demand, but mitochondrial Ca^2+^ overload leads to the MPT, which causes the disruption of mitochondrial membrane integrity, irreversible oxidative damage, and the loss of ATP production, finally resulting in cell death. This may be achieved by altering the redox state, decreasing energy demand, or supplying the cells with pharmacological inhibitors of the MPT, such as cyclophilin inhibitors [62] (see also below).

RETRACTED

### Inflammation

This phenomenon occurs very rapidly and is more robust during reperfusion. The inflammatory reaction of the blood vessels occurs immediately after vessel occlusion and induces the activation of platelets and endothelial cells. The expression of adhesion molecules including selectins, intercellular adhesion molecules, and vascular cell adhesion molecules is induced by the adhesion of neutrophils initially and then later monocytes to the endothelium. Brain ischemia induces an inflammatory reaction that leads to mitochondrial damage [63]. Activated leukocytes contribute to blood vessel occlusion, which disturbs vascular patency and releases proinflammatory cytokines, proteases, and ROS that induce vascular damage at the endothelial surface, leading to thrombus formation, vasospasm, and breakdown of the blood-brain barrier, further promoting the infiltration of leukocytes into the brain. Activation of microglia, which are the resident tissue macrophages, occurs within minutes of the onset of ischemia. After neuronal cell death, danger-associated molecular pattern molecules activate the pattern recognition receptors, including the Toll-like receptors expressed on microglia, and contribute to the inflammatory response in brain ischemia. Microglia also produce ROS that can cause mutations in mitochondrial DNA and damage the enzymes of the respiratory chain, leading to dysfunction of oxidative phosphorylation and increased ROS production [64]. The early inflammatory response therefore appears to induce the secondary failure of bioenergetic function.

### Molecular mechanisms of the mitochondrial permeability transition (MPT)

The MPT was traditionally considered to be mediated by the formation of an MPT pore, which is a dynamic complex of several proteins. This protein complex was proposed to be located at the contact sites between the inner and outer mitochondrial membranes, which are sites important for metabolic regulation as well as interaction with the cytosol, intermembrane space, and the matrix compartments [65, 66]. It is still unclear whether the elevation of mitochondrial matrix Ca^2+^ levels during ischemia is causally related to the neuronal cell death that occurs after cerebral ischemia. The current general hypothesis is that the MPT is formed by the voltage-dependent anion channel (VDAC or porin) of the outer membrane, the adenine nucleotide translocase (ANT) of the inner membrane, and cyclophilin D (CypD) located in the matrix compartment [66]. However, a recent gene deletion study has questioned the role of VDAC as an essential component and regulator of the MPT [67].

RETRACTED

The increased permeability of the inner mitochondrial membrane can also possibly be induced by the concerted action of other proteins such as the uncoupling proteins and the Tom/Tim transport system, as well as by the aggregation of misfolded membrane proteins. However, the proposed core components of the MPT pore, in particular ANT and CypD, are likely to be the proteins involved in the MPT phenomenon during calcium overload under pathophysiological conditions. Hansson et al. reported that adult-viable human brain and liver mitochondria possess an active CypD-sensitive mtPTP and that CypD inhibition plays an important role for neuroprotection [68–70].

In summary, the obligate molecular components of the MPT have not yet been resolved. Initially, there was the hypothesis that the MPT requires a complex consisting of the inner membrane protein ANT, the outer membrane component VDAC/porin, and the matrix modulator CypD.

### Critical role of the MPT in neurodegeneration

The loss of ATP; an increase in the levels of calcium, phosphate, and free fatty acids; and the generation of free radicals are key factors in inducing the MPT (Fig. 4). The proton gradient and the mitochondrial membrane potential (ΔΨm) are rapidly lost as the hydrogen ions extruded from the mitochondria by the electron transport chain rapidly fall back through the MPT pores, uncoupling oxidation of metabolic substrates and respiration from the phosphorylation of ADP. The consequences of the MPT are dramatic when the inner membrane rapidly becomes permeable to solutes of up to 1500 Da (Fig. 4). Importantly, this transition, if prolonged, can affect respiration in different ways according to the substrate being oxidized. Induction of the MPT in mitochondria energized with complex-I-linked substrates is followed by complete respiratory inhibition due to the loss of pyridine nucleotides [71, 72]. Induction of the MPT in mitochondria energized with complex-II-linked substrates is followed by uncoupling. The mitochondrial matrix is dense in proteins, and the induction of the MPT pores will result in an osmotic influx of water into the matrix, causing the inner membrane to unfold and expand, resulting in mitochondrial swelling, as well as causing the outer membrane to rupture, inducing the release of proapoptotic proteins such as cytochrome c [73, 74] and apoptosis-inducing factors Omi and Smac (Fig. 4). Prolonged and extensive MPT will lead to the termination of ATP production and necrotic cell death, if the energy balance cannot be compensated by anaerobic metabolism.

RETRACTED

### Calcineurin and cell death

Calcineurin was first discovered by Wang et al*.* in 1976 as an inhibitor of calmodulin (CaM)-dependent cyclic phosphodiesterase [75]. Calcineurin is abundantly distributed in the hippocampus, striatum, and cerebral cortex. Subcellularly, it is primarily found bound to the cell membrane or the cytoskeletal elements and is enriched in postsynaptic densities. Calcineurin is best known as being a target for the widely used immunosuppressive molecules cyclosporin-A (CsA) and tacrolimus (FK506) [76]. Under physiological conditions, the effects of calcineurin are greatly multifaceted, for example, it can dephosphorylate NMDA receptors, IP3 receptors, and ryanodine receptors, which are all relevant to the regulation of intracellular Ca^2+^ levels. Shibasaki et al*.* demonstrated the interaction between members of the antiapoptotic Bcl-2 protein family and calcineurin activity, indicating an important role for calcineurin in the regulation of apoptosis [77]. They furthermore demonstrated that calcineurin specifically participates in a Ca^2+^-inducible mechanism for apoptosis induction by regulating BAD (a proapoptotic Bcl-2 protein family member) phosphorylation [78] (see Fig. 4).

## Conclusions

Mechanisms of brain injury due to cardiac arrest and delayed neuronal death that occurs over hours to days after ROSC remain unknown. The pathophysiology of PCAS involves a complex cascade of molecular events, most of which are still unknown. Many lines of research evidence have shown that mitochondria suffer severe damage in response to ischemic injury. Mitochondrial dysfunction based on the MPT after reperfusion, particularly involving the calcineurin/immunophilin signal transduction pathway, appears to play a critical role in the induction of brain injury following cardiac arrest.

## Abbreviations

ACS: acute coronary syndrome
AMPA: α-amino-3-hydroxy-5-methylisoxazole-4-propionic acid
ANT: adenine nucleotide translocase
CsA: cyclosporin-A
FK506: tacrolimus
H_2_O_2_: hydrogen peroxide
MPT: mitochondrial permeability transition
NMDA: *N*-methyl-*D*-aspartate
O^2−^: superoxide anion
OH^−^: hydroxyl radical
OHCA: out-of-hospital cardiac arrest
PCAS: post-cardiac arrest syndrome
ROS: reactive oxygen species
ROSC: return of spontaneous circulation
VDAC: voltage-dependent anion channel
